The article "Bioinformatics Analysis of the Molecular Mechanism and Potential Treatment Target of Ankylosing Spondylitis" was published in 2021. Journal: Comput Math Methods Med.

# Bioinformatics Analysis of the Molecular Mechanism and Potential Treatment Target of Ankylosing Spondylitis

**DOI:** 10.1155/2021/7471291

**Published:** 2021-07-21

**Authors:** Fanyan Meng, Ningna Du, Daoming Xu, Li Kuai, Lanying Liu, Minning Xiu

**Affiliations:** ^1^Department of Acupuncture and Rehabilitation, Jiangsu Provincial Hospital of Traditional Chinese Medicine, China; ^2^Department of Nursing, Jiangsu Provincial Hospital of Traditional Chinese Medicine, 155 Hanzhong Road, Nanjing, China

## Abstract

Ankylosing spondylitis (AS) is an autoimmune disease that mainly affects the spinal joints, sacroiliac joints, and adjacent soft tissues. We conducted bioinformatics analysis to explore the molecular mechanism related to AS pathogenesis and uncover novel potential molecular targets for the treatment of AS. The profiles of GSE25101, containing gene expression data extracted from the blood of 16 AS patients and 16 matched controls, were acquired from the Gene Expression Omnibus (GEO) database. The background correction and standardization were carried out utilizing the transcript per million (TPM) method. After analysis of AS patients and the normal groups, we identified 199 differentially expressed genes (DEGs) with upregulation and 121 DEGs with downregulation by the limma R package. The results of the Kyoto Encyclopedia of Genes and Genomes (KEGG) pathway and Gene Ontology (GO) biological process enrichment analysis revealed that the DEGs with upregulation were mainly associated with spliceosome, ribosome, RNA-catabolic process, electron transport chain, etc. And the DEGs with downregulation primarily participated in T cell-associated pathways and processes. After analysis of the protein-protein interaction (PPI) network, our data revealed that the hub genes, comprising MRPL13, MRPL22, LSM3, COX7A2, COX7C, EP300, PTPRC, and CD4, could be the treatment targets in AS. Our data furnish new hints to uncover the features of AS and explore more promising treatment targets towards AS.

## 1. Background

Ankylosing spondylitis (AS), which mostly occurs in the sacroiliac joints, spine, and external joints (1), is a rheumatic immune disease with an incidence of 0.3% in China (2). AS patients are mostly young men (3). Most patients have early symptoms like dull pain in the waist, buttocks, and sacroiliac areas, later with complications in the heart, eyes, ears, and nervous system (4). The specific pathogenic mechanism of AS is not yet clear. It is only understood that genetic factors play major roles in AS pathogenesis (5). Besides, environmental, immune, metabolic, and other factors are also common causes of AS (6). Presently, AS cannot be completely cured. Most patients can be treated with nonsteroidal drugs and exercise. In severe cases, surgery is required (7). It should be noted that AS does not affect the survival of patients, but it will gradually ruin their lives (4). Therefore, to avoid the aggravation of AS patients, new treatment methods need to be developed as soon as possible.

The article "Bioinformatics Analysis of the Molecular Mechanism and Potential Treatment Target of Ankylosing Spondylitis" was published in 2021. Journal: Comput Math Methods Med.

Bioinformatics is a new interdisciplinary subject that takes computer as a tool to store, retrieve, and analyze biological information in the study of life sciences (8). At present, the research focus of bioinformatics is mainly embodied in genomics and proteomics (9), which is to analyze the biological information of the structure and function expressed in the sequence from the point of view of nucleic acid and protein sequences. Bioinformatics also plays an important role in the study of human diseases (10). Such as the establishment of disease-related bioinformatics database (11), isolation and identification of human genes and disease-related genes (12), and accelerating the development of gene drugs (13), these have an important and positive impact on the prevention and treatment of human diseases. We here executed bioinformatics analysis to investigate the molecular mechanism of AS pathogenesis and dig out the unclear details and probable treatments towards AS. GSE25101 was utilized to detect the differentially expressed genes (DEGs) in the specimens of AS patients and normal controls. Then, the molecular mechanism of AS was obtained after analyzing the pathway and functional enrichment. Finally, with the use of these DEGs, we established the protein-protein interaction (PPI) network to seek prospective genes in targeting AS.

## 2. Material and Methods

### 2.1. Data Source

GSE25101 (14), as the RNA expression profiles, was downloaded from the Gene Expression Omnibus database (GEO, https://www.ncbi.nlm.nih.gov/geo/) in NCBI. GSE25101 contained RNA expression data extracted from the blood of 16 AS patients and 16 matched controls using PAXgene tubes (15).

### 2.2. Data Preprocessing and the DEG Screening

The expression data of the GSE25101 data set was normalized by the transcript per million (TPM) method. Ensembl transcript IDs were transformed into the symbols of genes. The mean value was regarded as the expression level of genes if diverse probes were annotated to the same genes. Then, we utilized the limma R package to screen the DEGs between AS patients and normal control groups. The cut-off setting was *P* < 0.05 and ∣log_2_ fold change | >0.378511 based on the Benjamini and Hochberg (BH) procedure. Morpheus was applied to draw the heat map based on the website (https://software.broadinstitute.org/morpheus/).

The article "Bioinformatics Analysis of the Molecular Mechanism and Potential Treatment Target of Ankylosing Spondylitis" was published in 2021. Journal: Comput Math Methods Med.

### 2.3. Analysis of Pathway and Functional Enrichment

Metascape was applied to analyze the Kyoto Encyclopedia of Genes and Genomes (KEGG) pathway and Gene Ontology (GO) biological process enrichment (16) by accessing at https://metascape.org/gp/index.html#/main/step1. All genomic genes are thought of as enriched background. We obtained the top 20 significantly enriched terms with regard to the *P* values which were obtained on the basis of the accumulative hypergeometric distribution.

### 2.4. Analysis of the PPI Network

The Search Tool for the Retrieval of Interacting Genes (17) (STRING, https://string-db.org) was executed to analyze and visualize the PPI network of upregulated and downregulated DEGs. A medium confidence score > 0.400 indicated there was a great difference. Moreover, hub genes, as pivotal candidate genes with essential physiological regulatory use, were selected based on their degree of importance.

## 3. Results

### 3.1. Data Preprocessing and the DEG Screening

TPM was exploited to standardize the transcriptome expression data of the GSE126118 dataset. The limma R package was taken to screen the DEGs between AS patients and matched control groups. The volcano plot showed the identified DEGs (Figure 1(a)). According to the critical criteria of *P* value < 0.05 and ∣log_2_ (fold change) | >0.378511, 320 DEGs were screened. Among these, 199 DEGs were increased and 121 DEGs were decreased. In addition, we also constructed the gene expression heat map with color patterns to indicate the difference of gene expression existing in AS patients and normal groups (Figure 1(b)).

### 3.2. Analysis of Pathway and Functional Enrichment

Given the ontology sources, including KEGG pathways and GO biological processes, we analyzed pathways and functional enrichment of the DEGs by Metascape. All genes were regarded as the enrichment background. According to the calculated *P* values in the light of accumulative hypergeometric distribution, the top 20 with statistically obvious KEGG pathways and GO biological processes associated with upregulated and downregulated DEGs were presented in Figures 2 and 3, respectively. It could be observed that the DEGs with upregulation primarily participated in RNA- and protein-associated pathways, such as spliceosome, ribosome, oxidative phosphorylation, proteasome, RNA degradation, and protein export (Figure 2(a)). The enriched biological process of upregulated DEGs was related to energy production such as respiratory electron transport chain, oxidative phosphorylation, cytochrome c to oxygen mitochondrial ATP synthesis coupled electron transport, and ATP synthesis coupled electron transport (Figure 2(b)). The downregulated DEGs were enriched in pathways and processes associated with the immune response, especially Th17, Th1, and Th2 cell differentiation; T cell receptor signaling pathway; antigen processing and presentation; positive T cell selection; lymphocyte differentiation; lymphocyte activation touching upon the immune response; immune response-activating cell surface receptor signaling pathway; antigen receptor-mediated signaling pathway; T cell selection; and activation and differentiation (Figures 3(a) and 3(b)).

The article "Bioinformatics Analysis of the Molecular Mechanism and Potential Treatment Target of Ankylosing Spondylitis" was published in 2021. Journal: Comput Math Methods Med.

### 3.3. PPI Network Analysis

The STRING software for constructing the PPI network was utilized to investigate the interplay among the DEGs. Data from the STRING database revealed that these DEGs interacted with each other.  Figure 4 showed that the PPI network of upregulated DEGs was composed of 198 nodes and 734 edges. Among the 198 nodes, MRPL13 (degree = 26), LSM3 (degree = 25), COX7A2 (degree = 24), COX7C (degree = 24), and MRPL22 (degree = 23) were the top 5 significant hub node genes. Also, the PPI network of downregulated DEGs (Figure 5) contained 120 nodes and 159 edges. Among the 120 nodes, EP300 (degree = 15), PTPRC (degree = 15), and CD4 (degree = 14) were the top 3 significant hub node genes.

## 4. Discussion

AS is a complex disease that involves many factors (6). For patients with AS, there is currently no complete cure. The only way for patients to improve the poor prognosis is to actively cooperate with treatment and perform some rehabilitation exercises. Besides, early detection and early treatment are very necessary for patients. There is evidence showing that some lncRNAs are also involved in the development of AS. Some research shows that HLA-B27 may be involved in the pathogenesis (18). For example, Li et al. reported that the expression of lncRNA MEG 3 was downregulated in AS (19), which affected the length of the patient's hospital stay. Tan et al. proposed that the pathogenesis of AS might be related to insufficient autophagy and downregulation of lncRNA GAS 5, and lncRNA GAS 5 might have clinical application value (20). Our discovery gives a new hint of uncovering the traits of AS and exploiting a prospective target for AS treatment.

Our study attempted to explore the underlying mechanisms related to the AS. Public gene expression data from the GEO database GSE25101 were applied to analyze the data. To be first, we normalized the raw data and dug out the DEGs existing in AS patients and normal controls. Then, we performed the KEGG and GO analyses to detect these DEG-related pathways and biological processes. We identified 199 DEGs with increase and 121 DEGs with a reduction from a PPI network. The data of enrichment analysis revealed that the DEGs with upregulation majorly participated in the spliceosome, ribosome, RNA-catabolic process, electron transport chain, and so on. The DEGs with downregulation mostly took part in T cell-associated pathways and processes. Studies have shown that some new congenital or physical diseases are related to mutations in secondary spliceosome components (21), such as cerebellar ataxia, myelodysplastic syndrome, spondyloepiphyseal dysplasia tarda, amyotrophic lateral sclerosis, and spinal muscular atrophy. The generation of reactive oxygen species (ROS) by the mitochondrial electron transport chain (ETC) is thought to be important in the pathogenesis of neurodegenerative diseases such as the aging process and Parkinson's disease (22). The PPI network analysis revealed that MRPL13, MRPL22, LSM3, COX7A2, and COX7C were the hub upregulated genes in AS, and EP300, PTPRC, and CD4 were the hub genes with downregulation in AS.

The article "Bioinformatics Analysis of the Molecular Mechanism and Potential Treatment Target of Ankylosing Spondylitis" was published in 2021. Journal: Comput Math Methods Med.

Nuclear genes encode MRPL13 and MRPL22 which are the members of mitochondrial ribosomal proteins (MRPs). MRPL13 and MRPL22 are generated in the cytoplasm and then transported to mitochondria to assemble mitochondrial ribosomes (23). MRPs are essential for mitochondrial oxidative phosphorylation and exhibit crucially in regulating apoptosis-inducing factors (24). Aberrant MRP expressions will result in multiple dysregulations, such as disordered mitochondrial metabolism and dysfunctional cell (25). Here, we report abnormally expressed MRPs in AS.

LSM3, as a constituent of the precatalytic spliceosome, participates in the assembly of the spliceosome (26). It functions essentially in the process of pre-mRNA splicing as a part of the U4/U6-U5 tri-snRNP (27). Pre-mRNA splicing displays an essential role in the generation of mature mRNAs in eukaryotic cells to regulate gene expression (28). Combined with the enrichment analysis, our results suggested that the AS exhibited a relation with the spliceosome. COX7A2 and COX7C are the components of the cytochrome c oxidase (COX) which is the terminal enzyme of the mitochondrial respiratory chain. COX is responsible for catalyzing the reduction of oxygen to water, which is critical for energy production in all organisms (29). The COX-related pathway contains ATP synthesis, respiratory electron transport, heat production, and so on, consistent with our enrichment analysis.

Ep300 encodes a p300 transcriptional coactivator associated with adenovirus E1A (30). Histone acetyltransferase Ep300 mediates the modulation of transcription via remodeling chromatin, cell proliferation, and differentiation (31). Ep300 has also been reported as a coactivator of HIF1A (hypoxia-inducible factor 1 alpha) thus activating VEGF which is a hypoxia-induced gene (32). Diseases associated with EP300 contain Menke-Hennekam Syndrome 2 and Rubinstein-Taybi Syndrome 2 (33). Pathways related to EP300 contain regulating TP53 activity through acetylation and Nur77 signaling in the T cell. Protein Tyrosine Phosphatase Receptor Type C (PTPRC) belongs to the tyrosine phosphatase family, generally functioning as a regulator of several cellular processes, i.e., mitosis, cell proliferation and differentiation, and oncogenic transformation (34). PTPRC is shown to be a fundamental molecule in regulating T cell and B cell antigen receptor signaling (35). PTPRC-related signaling works via direct interaction with the antigen receptor complex or through motivating several kinases of the Src family. CD4 membrane glycoprotein, also named as the CD4 antigen, is encoded by the CD4 gene of T lymphocytes (36). Not only do T lymphocytes express CD4 genes, but also macrophages, B cells, granulocytes, and various regions of the brain do. The CD4 membrane glycoprotein along with T cell receptors works together as receptors to recognize antigens presented by antigen-presenting cells under the circumstance of class II MHC molecules (37). It can activate or enhance the early stage of T cell activation and exhibit as a central mediator of indirect neuronal damage in infectious and immune-mediated diseases of the central nervous system. To sum up, these three genes are associated with T cells which are consistent with our enrichment analysis of downregulated genes and could be the treatment targets.

The article "Bioinformatics Analysis of the Molecular Mechanism and Potential Treatment Target of Ankylosing Spondylitis" was published in 2021. Journal: Comput Math Methods Med.

The study has some limitations. The expression level of the hub gene in AS needs further verification. In the following study, we will collect clinical samples and determine the expression level of the hub gene through TaqMan Real-Time PCR. We will further explore the correlation between hub gene expression and clinical parameters (including clinical stage, age, and survival time).

## 5. Conclusion

This study used the bioinformatics method to analyze gene expression data of GSE25101 to unearth the considerable points and promising targets in AS treatment. In total, we screened 199 DEGs with upregulation and 121 DEGs with downregulation after analyzing AS patients and normal control ones. KEGG and GO enrichment analyses demonstrated that the upregulated DEGs were largely associated with spliceosome, ribosome, RNA-catabolic process, and electron transport chain. And the DEGs with downregulation were generally enriched in T cell-associated pathways and processes. PPI network analysis revealed that MRPL13, MRPL22, LSM3, COX7A2, COX7C, EP300, PTPRC, and CD4 were the hub genes in AS and could be the treatment targets. Our data furnish new hints to uncover the features of AS and explore more promising treatment targets towards AS. In the medical field, it has positive and important significance for the future treatment of AS.

The article "Bioinformatics Analysis of the Molecular Mechanism and Potential Treatment Target of Ankylosing Spondylitis" was published in 2021. Journal: Comput Math Methods Med.

## Figures and Tables

**Figure 1:** (a) Volcano plot and (b) heat map show the DEGs between AS patients and normal controls. Blue indicates low expression values, and red represents high expression values. G1 and G2 represent AS patients and the normal control group, respectively.

**Figure 2:** (a) KEGG pathway and (b) GO biological process enrichment analysis of upregulated DEGs using Metascape. The top 20 significantly enriched terms are presented.

**Figure 3:** (a) KEGG pathway and (b) GO biological process enrichment analysis of downregulated DEGs using Metascape. The top 20 significantly enriched terms are presented.

**Figure 4:** Analysis of the PPI network of the DEGs with upregulation by the STRING database. Circle and line represent the protein and interaction, respectively.

**Figure 5:** Analysis of the PPI network of the DEGs with downregulation by the STRING database. Circle and line represent the protein and interaction, respectively.

## Data Availability

The datasets used and/or analyzed during the current study are available from the corresponding author on reasonable request.
